The article "How to promote the balanced development of urban and rural China? Evidences from reallocating idle rural residential land of Zhejiang province, China" was retracted in 2025. Reasons: concerns about the results or conclusions; concerns about the peer review; concerns about the authorship.

# How to promote the balanced development of urban and rural China? Evidences from reallocating idle rural residential land of Zhejiang province, China

**DOI:** 10.1371/journal.pone.0287820

**Published:** 2023-06-29

**Authors:** Zhenhua Hu, Gaohui Song, Ziyue Hu, Bo Zhang, Ting Lin

**Affiliations:** 1 School of Business, Wenzhou University, Wenzhou, China; 2 Hangzhou Dianzi University, Hangzhou, China; 3 Centre for Applied Macroeconomic Analysis, Australian National University, Canberra, Australia; Shenzhen University, CHINA

## Abstract

As more attention is given to green and sustainable industries, an analysis of the industrial impacts on all aspects of life, including inclusive affluence, is gradually developing. Idle rural residential land is a valuable resource and an important factor in promoting sustainable development. Balanced urban and rural development contributes to inclusive prosperity, so understanding the relationship between industry and the balanced development of urban and rural can significantly impact social development. In China, achieving the balanced development requires narrowing the urban-rural income gap. This paper analyzed the impact of reallocating idle rural residential land on promoting the balanced development. The study found that industry development has a positive impact on the balanced development, with a regression coefficient of 1.478. Regions with higher industry indices in counties had better outcomes regarding the balanced development. When the development of rural industry derived from idle residential land was in good condition, the effect increased by 3.326 percentage. The results showed heterogeneity, with the regression coefficient of industry development on the balanced development in county-level cities being 0.498 larger than in urban areas. In summary, the reallocation of idle residential land can promote sustainable development, increase residents’ income, and improve overall regional economic development. The results are applicable to the comprehensive reallocation of rural land resources.

## 1. Introduction

The efficient utilization of resources, particularly idle and abandoned ones, is crucial for the sustainable development of both the economy and society, as well as the well-being of humanity. Numerous countries have undertaken efforts to promote resource recycling, and explore the potential value of underutilized land, using market mechanisms, active engagement from different stakeholders, and effective resource management. China, too, has embarked on this journey, with a focus on Idle Rural Residential Land (IRRL), underlining the central importance of developing rural industries and bridging the urban-rural divide.

Currently, there is a growing national effort to bridge the urban-rural divide. Several studies have focused on inclusive affluence, including connotation [1], addressing measures [2–4], and corresponding experience [5, 6]. To improve the village economy, full advantage of rural culture and resources is being taken under the guidance of the theory of regional integration, with the development of leisure industries [7–10]. Empirical analyses by some scholars have shown that city-biased policies, infrastructure construction, and industrial development have an important influence on narrowing the urban-rural gap [11]. Additionally, the improvement of rural education levels can significantly affect economic development [12]).

China has approximately 2,844 county-level administrative divisions, and the county economy contributes approximately 53% to China’s GDP. Serving as a vital junction between urban and rural areas, the county economy plays an integral role in promoting social and economic integration. Zhang Jian, who recognized the potential of county economy as early as 1986, believed that developing tertiary industries in counties and reallocating IRRL would result in industry growth, employment opportunities, and ultimately, shared prosperity among rural residents [13]. The correlation between industry and urban-rural balanced development, particularly in relation to IRRL, is a contentious issue.

This paper aimed to digitally characterize the amount of inclusive affluence promoted by industrial development driven by idle rural land. The innovation of this paper was reflected in that it measures the balanced development of urban and rural areas by constructing the inclusive affluence index, and verifies that the regional industrial development and rural industry development under the reuse of IRRL played a positive role in promoting the balanced development of urban and rural areas. The significance of this paper lied in quantifying the economic value with certain values and providing economic impetus for promoting the utilization of rural idle land. Additionally, it provided a new idea for researching the reallocation of idle land resources.

## 2. Materials and methods

### 2.1 Study area and data

Zhejiang Province is situated on China’s southeast coast, spanning an area of 101,800 square kilometers and home to a population of 50.3891 million. The province’s agriculture, forestry, animal husbandry, and fishery industries have generated an added value of 213.53 billion yuan, while rural leisure agriculture has seen significant growth, with a total output value of 44.27 billion yuan and hosting up to 250 million tourists. Over the past five years, there has been significant development in rural housing land, with 91,000 hectares of existing land, totaling 9.95 million cases. Roughly 7.09 million homestead registrations, taking up an area of approximately 64,000 hectares, accounted for around 71% of completed approvals. The integration of real estate has also seen promising results, with an IRRL of about 530,000, accounting for 4.36% of the total IRRL and 32.02% of which have already undergone transfers.

Zhejiang Province has the comparative advantages of small urban-rural income gap, high degree of balanced regional development and good level of affluence. It has a variety of landforms including plains, basins, islands and hills, which give birth to diverse urban and rural types and development patterns. It is a typical representative of China’s high-quality construction and common prosperity demonstration area. Fig 1 shows that the per capita disposable income of urban and rural residents is increasing year by year, and the rate of increase of rural residents is faster than that of urban residents, which ultimately further narrows the gap between urban and rural per capita disposable income, indicating that the Gini coefficient is also narrowing. In addition, Fig 2 proves that the tourism industry of Zhejiang is in good condition. Therefore, considering the case of Zhejiang Province offers valuable insight into the relationship between regional industry development and urban-rural balanced development stemming from the utilization of IRRL.

**Fig 1:** 2015–2020 urban-rural income gap in Zhejiang Province.

**Fig 2:** 2015–2019 rural tourism and total revenue in Zhejiang Province.

Zhejiang Province comprises of 11 prefecture-level cities and a total of 89 county-level administrative regions. However, the county-level data was found to be partially missing or discontinuous due to the establishment or merger of some cities from 2015 to 2019. Nonetheless, our sample was still considered relatively representative as it covered more than 70% of the county-level cities. The data utilized in this study were sourced from the Zhejiang Statistical Yearbook (ZSY, 2016–2020) as well as various Urban Statistical Yearbooks. It is worth noting that we conducted standardized processing of data to eliminate errors and ensure accurate results.

### 2.2 Theory analysis and research hypothesis

#### 2.2.1 The promotion of regional industrial development contributes to urban-rural balanced development

Industry is a crucial element of economic progress and serves as the bedrock for achieving inclusive prosperity. Considering multiple factors, the article narrowed down to two primary factors influencing the relationship between industry growth and urban-rural balanced development.

The first key factor in achieving prosperity is industry growth. A stable industrial foundation and an optimized industrial structure are essential for high-speed and efficient growth of the regional economy. Building a modern industrial system and undertaking the transfer of industries from developed areas can strengthen the industrial foundation and lead to economic growth in less developed areas [14]. Industry development can also promote employment and increase the wages of the labor force, thus significantly improving the sustainable livelihood of villagers [15–18].

The second crucial factor is inclusive affluence. Industry development can promote regional balanced development as big cities radiate to surrounding cities [19]. According to the theory of regional economy, the interregional flow of factors of production tends to converge, leading to the promotion of human capital, technology, land, capital, and other factors of production. Adjusting income distribution by factors of production, promoting the rational allocation of regional resources, and equally accessing wealth can help improve people’s well-being and acquisition. This meant that industry development not only helped increase wealth but can also perfected the efficiency of sharing. Hypothesis 1 was put forward in this context.

Hypothesis 1: Regional industrial development had a positive effect on the urban-rural balanced development and inclusive affluence.

#### 2.2.2 Rural industries developed through IRRL played a significant role in promoting urban-rural balanced development

The thriving rural industry played a pivotal role in the county’s economic growth and rejuvenation [8, 20]. With the increasing diversification of the agricultural industry, rural tourism has positively impacted the income levels of villagers [21, 22]. According to the Tourism Driven Growth theory, tourism promotes economic development by generating employment opportunities, investments, and consumption [23]. Rural tourism, including agro-tourism, leisure tourism, and ecological tourism, is regarded as a cornerstone for the innovation of the agricultural structure. Therefore, the vast rural resources serve as valuable assets and capital for rural tourism, essential for its sustainable development [24–26].Eliminating the urban-rural gap and boosting rural resident income is crucial, given the existence of wage rigidity. This would hasten the adjustment of the rural industrial structure [27], further fuelling the rural economy. By utilizing rural resources, various industries such as agrotourism, courtyard economy, and family homestay can stimulate rural development effectively [28] Hence, this research aimed to optimize the industrial structure’s layout and promoted industrial development in the county [29–32].

Additionally, China’s unique national conditions enabled the active reallocation of rural idle resources, through a combination of internal hierarchical governance and market management strategies such as the Industrialization of Rural Residential Land (IRRL) and promoting rural industry to improve land function. This approach helped alleviate pressure on urban employment and minimize economic risks. Therefore, the development of the rural industry, through coordinated efforts from various industries, was crucial in achieving inclusive prosperity. As a result, hypothesis 2 was put forward.

Hypothesis 2: Rural industry growth had a positive effect on the promotion of regional industry growth to urban-rural balanced development.

The framework was illustrated in Fig 3.

**Fig 3:** Theoretical framework.

### 2.3 Methods

#### 2.3.1 Calculating the Inclusive Affluence Index (IAI) based on EW and PCA

The Entropy Weight (EW) method was chosen to objectively measure the evaluation index, while the Principal Component Analysis (PCA) was utilized to eliminate the mutual influence of evaluation indices and provide precise information. The Inclusive Affluence Index (IAI) was chosen to represent the degree of balanced urban and rural development. Thus, the IAI was calculated more accurately and objectively using the EW and PCA methods. The following formula and approach were adopted.

Firstly, each index *X* = {*X*_1_, *X*_2_, *X*_3_, ⋯ *X*_*m*_} was de-dimensioned. Supposing that *m* indicators are given. And *X_i_* = {*x*_1_, *x*_2_, *x*_3_, ⋯ *x*_*n*_}.

Secondly, *Y* = {*Y*_1_, *Y*_2_, *Y*_3_, ⋯ *Y*_*m*_} represented standardized value of each index data.


$$Y_{ij}=\frac{X_{ij}-\min\left(X_{i}\right)}{\max\left(X_{i}\right)-\min\left(X_{i}\right)},\;\left(\text{Positive}\;\text{index}\right)$$ (1)

$$Y_{ij}=\frac{\min\left(X_{i}\right)-X_{ij}}{\max\left(X_{i}\right)-\min\left(X_{i}\right)},\;\left(\text{Negative}\;\text{index}\right)$$ (2)

Thirdly, the entropy of information for each index was computed. Assuming that there were *m* secondary indicators for a primary indicator, and *n* years of data were collected, which was represented as a matrix. For each index, the proportion of each year’s value in the total value was calculated. The formulas used for computation were as Eq 3.


$$p_{ij}=\frac{Y_{ij}}{\sum_{i=1}^{n}Y_{ij}}(i=1,2,\cdots n;j=1,2,\cdots m)$$ (3)

The *E*_*j*_ represented the information entropy value, then

$$E_{j}=-\ln{\left(n\right)}^{-1}\sum_{i=1}^{n}p_{ij}\;\ln\;p_{ij}$$ (4)

Fourthly, the weights of each index were calculated.


$$w_{j}=\frac{1-E_{j}}{m-\sum_{}^{}E_{j}}$$ (5)

Finally, the comprehensive measurement results of variables were presented.


$$s_{i}=\sum_{j=1}^{m}w_{j}\times x_{ij}$$ (6)

Based on the above results, the following formula was obtained by PCA.


F1=0.693×affluence+0.693×sharing (7)

F2=0.722×affluence−0.722×sharing (8)

IAI=(0.52/1.0)×F1+(0.48/1.0)×F2 (9)

Where *F*1 and *F*2 respectively referred to the two principal component factors in the Principal Component Analysis, and *IAI* represented the Inclusive Affluence Index (IAI). For this study, a higher IAI indicated better the urban-rural balanced development. Stemming from the literature review, this study defined the inclusive affluence as “affluence” and “sharing”, then selected the following indicators was shown Tables A1 and A2 in S1 Appendix [33, 34]

#### 2.3.2 Calculating the Regional Industry Index (RII) based on EW and PCA

Similarly, this paper also selected various indicators to calculate the Regional Industry Index (RII) through EW and PCA. The specific calculation formula was shown in 2.3.1. And the results were given in Table A3 in the S1 Appendix.

#### 2.3.3 Constructing panel attribution-value model

In addition to the methods mentioned above, the article primarily employs the empirical approach. Specifically, the Attribution-Value Model was utilized to examine how one economic variable impacts another and how the effect is moderated by an additional variable. This widely-used measurement method in economic analysis considers the moderating variable as either positively or negatively affecting the relationship between the original variables. For this study, the regional industry development was seen as playing a crucial role in bolstering the economic condition, and ultimately promoting inclusive affluence. Building on previous research conducted by Yang [32, 35], the panel Attribution-Value Model was cautiously constructed in accordance with the research hypothesis as follows:

$$IAI_{it}=\beta_{0}+\beta_{1}RII_{it}+\sum \beta_{it}control_{it}+\varepsilon_{it}$$ (10)

$$IAI_{it}=\beta_{0}+\beta_{1}RII_{it}+\beta_{2}DRI_{it}+\beta_{1}RII_{it}\times DRI_{it}+\sum \beta_{it}control_{it}+\varepsilon_{it}$$ (11)

where *IAI*_*it*_ represented the realization of the inclusive affluence of *i* county and city in the *t* year, *RII*_*it*_ represented the regional industry development of *i* county and city in the *t* year, *DRI*_*it*_ represented the rural industry development of *i* county and city in the *t* year, *control*_*it*_ represented the control variable, *β*_1_ was the regression coefficient of the core independent variable, *β*_*it*_ represented the regression coefficients of the control variable, *ε*_*it*_ was the random disturbance term. And control variables mainly included financial market perfection, fiscal autonomy, population density, labor mobility, the proportion of welfare expenditure, per capita GDP, and so on. The regional and year dummy variables of Zhejiang Province were included to reduce the problem of missing variables among regions.

Assume *t* = 5 and *i* = 63 in this paper. And the data were panel data integrated with continuous cross-sectional data and time series data which could verify the accuracy of the above hypothesis more comprehensively. Generally speaking, the higher the significance of regression coefficient between variables, the greater the correlation.

## 3. Results

### 3.1 The description of parameter

The dependent variable was defined as IAI, while the explanatory variable was composed of RII and DRI. To address missing variables among regions, regional and year dummy variables for Zhejiang Province were also included.

Table 1 provided an overview of the descriptive statistics for all variables. The study found that the IAI had a greater level of volatility than the regional industry index. Specifically, the mean value of the IAI was 0.907 with a standard deviation of 1.161, indicating a higher level of fluctuation. The regional industry index, on the other hand, had a mean value of 0.068 with a standard deviation of 0.047. This suggests that the reuse of idle homesteads had a relatively small impact on the fluctuation of the RII.

**Table 1:** Descriptive statistics.

Variables		Abbreviation	Computing method	Mean	SD
Explained variable	the Inclusive Affluence Index	IAI	Entropy value method and Principal Component Analysis	0.907	1.161
explanatory variable	The Regional Industry Index	RII	Entropy value method	0.883	0.780
Moderating variable	The Development of Rural Industries	DRI	GDP of primary industry/GDP of the region	0.068	0.047
Control variables	Perfection of financial markets	FIN	the ratio of the balance of residential deposits and loans /GDP	2.178	3.883
	Financial autonomy	FEN	Total fiscal revenue/total fiscal expenditure	0.587	0.261
	Population density	PD	Land gross area/resident population	0.082	0.168
	Labor mobility	LM	2 &3 industry labor number/first industry labor force	2.046	6.236
	Per capita welfare expenditure	welfare	Total welfare expenditure / resident population in the area	0.524	0.813
	per capita GNP	lngnp	GDP/resident population	11.175	0.384

### 3.2 Regional Industry Index (RII) promoted the inclusive affluence

Revised benchmark regression was applied due to the presence of heteroscedasticity and sequence autocorrelation between variables even though cross-sectional autocorrelation was not observed. The estimated results of the model are presented in Table 2.

**Table 2:** Benchmark regression results.

Independent variables	(1)	(2)	(3)	(4)
RII	1.375*** (14.65)	1.426*** (20.66)	1.463*** (20.72)	1.478*** (23.44)
FIN		-0.0159*** (-3.18)		-0.0179*** (-2.86)
FEN		0.0323 (0.47)		-0.336 (-0.85)
PD		0.453*** (3.04)		0.0138 (0.06)
LM		-0.0314*** (-6.62)		-0.0329*** (-6.79)
welfare		0.00417 (0.18)		0.0721 (1.26)
DRI		2.084*** (5.04)		2.336 (0.69)
lngnp		14.33*** (5.28)		0.246* (1.87)
lngnp^2^		-0.660*** (-5.34)		
constant	-0.388*** (-5.57)	-78.13*** (-5.25)	-0.442*** (-7.58)	-3.096* (-1.99)
year	no	no	yes	yes
resident	no	no	yes	yes
R-squared	0.9321	0.9635	0.9333	0.9388
robustness	yes	yes	yes	yes
sample	315	315	315	315

Notes: Standard errors were in parentheses.

* p<0.1

** p<0.05

*** p<0.01.

The comparison results indicated that the positive impact of industry development on the realization of inclusive affluence was significant at the 1% significance level whether or not control variables were introduced, supporting hypothesis 1. After introducing control variables, both financial market perfection and labor mobility index had significant negative effects on inclusive affluence. Per capita GDP displayed an inverted U-shaped effect on the IAI. Specifically, the regression analysis of industry development in column (3) demonstrated that industry development had a significant positive effect on IAI with a regression coefficient of 1.463. After introducing control variables in column (4), the positive regression coefficient of industry development on inclusive affluence increased to 1.478, indicating that higher DRI in counties was correlated with better realization of inclusive affluence. The robustness of results was confirmed by the regression analyses in columns (1) and (2). According to column (2), county-level industry development could significantly promote inclusive affluence by 1.426 even when other conditions remained unchanged. This may be attributed to good industry development leading to improved income and employment, as well as meeting the need for basic public services, education investment, infrastructure construction, and other dimensions of social security, effectively enhancing the affluence and sharing satisfaction of residents.

Furthermore, the study found that different control variables had varying effects on inclusive affluence. Fiscal autonomy, per capita welfare expenditure, and rural industry development were all positively correlated with inclusive affluence. Meanwhile, financial market perfection and labor mobility index had minor negative effects. This was surprising, as financial market perfection was expected to have a positive impact on inclusive affluence. However, the variable was measured using the ratio of residential deposits, loans, and GDP which may have been biased. In our initial data, residential loans were higher than deposits, and the higher this ratio, the higher the chance of non-performing loans in the market. This could explain the negative effect, however, future research could optimize this variable. The rural-urban labor mobility index measured the proportion of the labor force in the secondary and tertiary industries. The smaller the primary industry’s labor force, the more agricultural employment, the fuller the rural labor force basis, and the greater the development potential. Since the Inclusive Affluence Index (IAI) included affluence and sharing, the urban and rural labor flow index hindered inclusive affluence. Moreover, per capita GDP had a significant inverted U-shaped effect on inclusive affluence, indicating that promoting per capita GDP above the critical value would weaken inclusive affluence. The higher the value of per capita GDP before this critical value, the better the situation of inclusive affluence, and beyond this value, the more the inclusive affluence would be weakened. Since inclusive affluence considers urban-rural income gaps being important indicators, economic development could lead to a widening of the income gap and inhibit the inclusive affluence at a certain point.

### 3.3 The development of rural industries (DRI) has a significant positive moderating effect on the RII and IAI

The findings suggested that regional industry development played a crucial role in promoting inclusive affluence by absorbing labor, alleviating urban housing and employment pressure, and supporting the growth of urban industries. To examine whether rural industries positively foster or negatively hinder regional industries in promoting inclusive affluence, this study used rural industry development as a moderating variable. The results of the moderated regression analysis, presented in Table 3, demonstrated that the interaction term between regional industry development and rural industry development had a significant positive effect on the IAI, as indicated by a regression coefficient of 3.326. This implied that rural industry development enhanced the impact of regional industrial development on promoting inclusive affluence. Specifically, when the primary industry was well-developed, the effect of industry development on inclusive affluence could increase by 3.326%. These findings underscored the significance of rural industry development in promoting county industry growth and achieving inclusive affluence. Additionally, the results of columns (2) and (4) supported the robustness of the moderating effects.

**Table 3:** Results of moderating.

Variable	(1)	(2)	(3)	(4)
RII	1.480*** (23.56)	1.069*** (19.30)	1.165*** (13.40)	1.163*** (39.73)
RII×DRI		3.906*** (8.44)	3.326*** (4.80)	3.322*** (11.69)
DRI		-2.822*** (-4.88)	-4.246* (-1.85)	-2.924** (-3.97)
FIN	-0.0178*** (-2.88)	-0.00844*** (-2.70)	-0.0105*** (-3.30)	-0.0108* (-2.52)
FEN	-0.334 (-0.84)	-0.00328 (-0.06)	0.0710 (0.25)	0.0793 (0.32)
PD	0.0350 (0.16)	0.126 (0.91)	-0.0362 (-0.17)	-0.0616 (-0.51)
LM	-0.0328*** (-6.81)	-0.0289*** (-6.27)	-0.0309*** (-6.50)	-0.0311*** (-13.41)
welfare	0.0672 (1.19)	0.0496* (1.67)	0.0794 (1.45)	0.0870** (4.24)
lngnp	0.206** (2.02)	-0.221*** (-4.26)	0.0197 (0.21)	-0.0269 (-0.45)
constant	-2.477** (-2.26)	2.353*** (3.98)	-0.322 (-0.27)	0.0966 (0.12)
year	yes	no	yes	No
resident	yes	no	yes	yes
R-squared	0.9364	0.9767	0.9673	0.9852
robustness	yes	yes	yes	yes
sample	315	315	315	315

Notes: Standard errors were in parentheses.

* p<0.1

*** p<0.01.

Rural revitalization has played a pivotal role in China’s economic development. The agricultural sector is the foundation on which rural revitalization is built. The country is grappling with the issue of abundant unused rural residential land, and a key solution is to promote the mutually beneficial integration of residential land and rural industries, this approach would foster rural revitalization and inclusive prosperity. In recent years, the national government has made significant investments to improve rural infrastructure such as roads, water, electricity, gas, and broadband, which has yielded positive results. Under the banner of the "new productive forces" strategy, early initiative by rural village collectives to reallocate unused rural residential land have paved the way for ecological civilization and rural revitalization, ultimately leading to the optimization and upgrading of the country’s industrial structure.

### 3.4 The heterogeneity and regional dynamic evolution of RII and IAI

While the regression results presented a linear relationship, there may be heterogeneity issues to consider. The disparities in industry development and inclusive affluence between urban and surrounding cities can significantly impact the results. The effect of industry development on "affluence" was more direct than on "sharing". Therefore, a heterogeneity analysis of 11 of the 63 cities in the urban area, separated from 52 counties, was conducted to verify the existence of regional heterogeneity.

The economic development and public service gap in urban areas were different from those in surrounding county-level cities. Urban areas generally had a higher economic development level and population density, which leaded to a better realization of inclusive affluence. The impact of industry development on the urban-rural balanced development was different on the city and county. This article analyzed in detail the two indexes that influenced the degree of inclusive affluence.

The results of the heterogeneity analysis (Table 4) showed that, under the condition that other factors remained the same, the regression coefficient of industry development to the inclusive affluence of county-level cities was 0.498 larger than that of urban areas. This indicated that in the same conditions, a unit change in the industry index would improve county-level affluence by 1.583 and urban affluence by 1.085, which further confirmed the robustness of the analysis results.

**Table 4:** Heterogeneity results.

variable	Regional heterogeneity		Replace the explained variable		
	52 counties	11 downtown	IAI	affluence	sharing
RII	1.583*** (129.56)	1.085*** (26.76)	1.428*** (20.41)	2.020*** (20.31)	0.00793 (0.25)
control	yes	yes	yes	yes	yes
resident	yes	yes	yes	yes	yes
year	yes	yes	yes	yes	yes
R-squared	0.9813	0.9875	0.9636	0.9632	0.1157
sample	260	55	315	315	315

Notes: Standard errors were in parentheses.

*** p<0.01.

After the replacement of explained variables, it was found that industry development played a more significant role in promoting "affluence" than in promoting "sharing" because industry development directly affected social wealth and indirectly affected social distribution.

In summary, there is a strong correlation between regional industrial development and inclusive prosperity. Notably, the correlation varied depending on the level of the city and the category of inclusive affluence. Therefore, these results not only supported the conclusions drawn in the article, but also provided a basis for future research on the relationship between rural industry development and inclusive affluence.

## 4. Discussion

### 4.1 The value of this paper

The significance of this paper was to explore the path to achieving the urban-rural balanced development and inclusive affluence through the reallocation of idle homesteads. This paper followed the industry perspective and employs the IAI and RII as main research methods for quantitative analysis of regional industry development, which was consistent with existing literature. However, unlike previous studies that primarily utilized questionnaire survey data [15, 22, 36], this paper used statistical yearbook data for empirical analysis, which was a more objective and innovative approach. Furthermore, the research topic aligned with the current social and economic development in Zhejiang Province, China. By quantifying the role of industry development in promoting the urban-rural balanced development and inclusive prosperity through the IRRL, this study provided compelling evidence for the development of relevant policies in China.

### 4.2 Reasons for selecting indicators

Compared to other scholars, those who measured the IAI and the RII emphasized the importance of objectivity and feasibility in selecting indices, leading them to prefer the Entropy Weight method [19, 21, 33, 34]. Although there was no standardized definition of the IAI, this paper drew from existing literature and utilized a credible set of indicators for its analysis. For instance, in terms of inclusive affluence, most indicator attributions were based on references, apart from urbanization and the elasticity of per capita income growth. The former was included because of the potential for rural people to earn higher wages and income in urban settings, while the latter was included to capture the impact of greater disposable incomes on fair social welfare. While the indicator system was not perfect, this study utilized scientific research and computing methods to refine its measurements (Table A1 in S1 Appendix).

To analyze regional industry development, this study relied on RII to measure the strength of industry development at the county level, using regional employment rates, real economic output value, import and export trade, industrial structure reorganization, and upgrading to reflect the overall economic strength of industry development (Tables A2 and A3 in S1 Appendix). It was noteworthy that industrial structural transformation and upgrading had a significant impact on regional economic development strength through industry-city linkage and economic growth effects [18]. Thus, a higher RII score indicated better regional industry development. For rural industry development, this paper selected the primary industry’s GDP proportion as a representative indicator. The primary industry includes agriculture, forestry, animal husbandry, and fishing, as well as the service industry. The rationale behind this selection was the inclusion of rural tourism, which was distinct from other kinds of tourism supporting agriculture, farmers, and rural life [37], but still closely tied to the primary industry.

### 4.3 The application of IRRL

Agriculture, rural areas, and villagers have always been a focus in China. It is of great significance to consolidate the foundation of rural industry development for the construction of a beautiful countryside in the long-term goal of China’s inclusive affluence construction. The fourth chapter concluded that regional industry development may effectively promoted the urban-rural balanced development, and the rural industry development derived from the reuse of IRRL positively promoted industrial development towards inclusive affluence. According to the Ministry of Agriculture and Rural Affairs of Zhejiang Province and the Survey of Inclusive Affluence in Zhejiang Province, Zhejiang province has actively explored the development of the regional overall industry and rural industry to promote the realization of the goal of the urban-rural balanced development and inclusive affluence.

Currently, there are 21,190 idle agricultural houses in Taizhou, among which 58.1% have completed the transfer, and 20.1% have the intention to transfer. By the beginning of 2019, Shaoxing City had completed the circulation of 10,585 IRRL through various plans such as the "Activation Plan of Idle Agricultural Houses", "Rural Mortgage", and "Posthouse Loan". In addition, more than 800 corresponding development and construction projects were introduced, which promoted the employment of more than 10,000 farmers and significantly increased the property income of village collectives and farmers. Special network promotion platforms such as "Township Road Network" in Shangyu, "Homesick Network" in Keqiao, and "Shared Courtyard" in Xinchang had promoted and completed the transfer of 2,937 and 1,397 IRRL.

The conclusion of the fourth chapter was consistent with the above social reality. On the other hand, the development of regional and rural industries was a good way to achieve the urban-rural balanced development. The development of the rural leisure industry under the reuse of IRRL not only promoted rural development but also promoted regional collaborative development and inclusive affluence [38].

## 5. Conclusions

In the process of urbanization, the number of rural migrant workers and IRRL was increasing significantly. Researchers paid more attention to this phenomenon. Most scholars only conducted quantitative or qualitative analysis of economic benefits brought by the reallocation of IRRL through small-scale questionnaire surveys, while relatively few conducted quantitative analysis from the macro level. To fill the above gaps in the study, this paper constructed a panel Attribution-Value Model based on the data index of 63 county-level cities in Zhejiang province over the past 5 years to empirically analyze and test the effect of industry development on the urban-rural balanced development. The following conclusions were drawn from the study: Firstly, regional industry development had a significant promoting effect on the realization of inclusive affluence. This study showed that the positive regression coefficient of industry development on the urban-rural balanced development was 1.478. Secondly, integrated rural industry development based on agriculture may significantly amplify the positive effect of industry development on the urban-rural balanced development, when the development of rural industry derived from IRRL was in good condition, the effect could be increased by 3.326%. Thirdly, heterogeneity analysis indicated that the effect of county industry development on the urban-rural balanced development was significantly greater than that of urban areas. Additionally, industry development could significantly improve the level of prosperity of residents, but the positive effect on sharing was not significant. In other words, if other conditions remain consistent, the regional industry index changed one unit, and county and urban affluence would improve by 1.583 and 1.085, respectively.

There were some limitations to this article. The study could only analyze the problem using limited data and did not consider the policy effect. The measures of IAI lacked a spiritual dimension. The industry developed by using idle homesteads was only a part of the rural industry, so this study may have some bias. However, the research results conform to economic development. In the future, follow-up research should construct a more scientific and comprehensive index system to evaluate inclusive affluence. Researchers could select data from a longer period for discussion, especially by adding consideration for policy impacts. Additionally, while protecting the vested interests of farmers, it is important to investigate the mechanism and cultivate patterns for further development of the joint IRRL and rural leisure industry.

## Supporting information

S1 Appendix (DOCX)

S1 Data (XLS)
